# Determinants of recommended antenatal care visits among pregnant women in Ethiopia: a generalized linear mixed-effects modeling

**DOI:** 10.1186/s12884-022-05213-w

**Published:** 2022-11-23

**Authors:** Hiwotie Getaneh Ayalew, Kibir Temesgen Asefa, Alemneh Mekuriaw Liyew

**Affiliations:** 1 Department of midwifery, school of nursing and midwifery, college of medicine and health sciences, Wollo University, Dessie, Ethiopia; 2 Department of Epidemiology and Biostatistics, Institute of Public Health, College of Medicine and Health Sciences, University of Gondar, Gondar, Ethiopia

**Keywords:** Antenatal care visit, Pregnancy, Generalized linear mixed-effects model, Ethiopia

## Abstract

**Background:**

Although antenatal care has the potential role to reduce maternal and child morbidity and mortality, utilization of a recommended number of antenatal care visits is still low in Ethiopia. Therefore, this study aimed to assess the determinants of recommended antenatal care visits in Ethiopia.

**Method:**

Data from the 2019 mini-Ethiopian demographic and health survey (MEDHS) was used for this study. A total of 3916 women who gave birth 5 years preceding the MEDHS were included. A generalized linear mixed-effects (mixed-effects logistic regression) model was used to identify the determinants of recommended antenatal care service utilization. Finally, the adjusted odds ratio with a 95% confidence interval and random effects were reported.

**Results:**

In the generalized linear mixed-effects model, women with primary education (AOR = 1.55, 95%CI 1.22–2.01), secondary and above education (AOR = 5.12, 95%CI 2.80–8.16), women from the middle (AOR = 1.25, 95%CI 1.01–1.71) and rich wealth index (AOR = 1.54, 95%CI 1.12–2.25), women who were exposed to media (AOR = 1.23,95%CI 1.01–1.57) and who use contraception (AOR = 1.45 95%CI 1.25–2.03), had higher odds of recommended antenatal care service utilization.

**Conclusion:**

In this study, factors like maternal educational status, media exposure, wealth index and history of contraceptive utilization were significantly associated with recommended ANC visits in Ethiopia. Therefore, encouraging women for contraceptive service utilization, consulting women to be exposed to media and improving women’s wealth status will help to have recommended number of ANC visits by pregnant women in Ethiopia.

## Background

Antenatal care (ANC) is healthcare service provided to pregnant women at health institution by skilled healthcare providers. It is provided throughout pregnancy to ensure better maternal and neonatal outcomes through risk identification, prevention and management of pregnancy-related or concurrent diseases [1]. It has the potential role to reduce maternal and neonatal morbidity and mortality and then improve neonatal and maternal health [2–6]. The ANC visit reduces the risk of neonatal mortality by 34% in sub-Saharan Africa [5]. Similarly, having adequate number of ANC visits reduces occurrence of maternal and neonatal complications. For instance, having four or more ANC visits can reduce about 81.2, 61.3, 52.4 and 46.5% risk of having postpartum hemorrhage, early neonatal death, preterm labor and low-birth-weight, respectively [6]. In general, having adequate antenatal care visits is best strategy to minimize the adverse pregnancy outcomes [7].

Globally, about 90% of pregnant women access antenatal care with skilled health personnel at least once and 57% receive at least four antenatal care visits. In countries with the highest rates of maternal mortality, like Africa and Asia, even fewer women received at least four antenatal care visits, 53 and 49% respectively [8, 9]. Lack of relevant and high-quality antenatal care services is a major concern in sub-Saharan Africa [10].

Ethiopia is part of sub-Saharan African countries and one of the countries with the highest maternal mortality ratios in developing countries [9]. The main causes of maternal mortality in Ethiopia include postpartum hemorrhage, sepsis, pre-eclampsia, eclampsia and birthing complications [11]. Even if most of these causes are preventable, many women often do not have access to evidence-based interventions such as antenatal care (ANC) services during pregnancy, due to poverty, lack of information, and cultural practices [12]. According to recent evidence from the Mini Ethiopian demographic health survey, only 43% of pregnant women had attended at list four ANC visits [13]. Thus, having antenatal care visits at recommended level (at least four visits during pregnancy) is still a major concern in Ethiopia.

In the previous studies, education level, employment status, marital status [14–16], ,occupation, residence, distance to the health facility [17], age, residence parity, and geographic location were identified as determinants of recommended ANC visits [15, 18–20]. However, the previous studies used traditional models and fail to account the random effects on the outcome variable. Generalized linear mixed effects model is a robust model which produces the reliable estimates for fixed effects by adjusting random effects [21, 22]. As to our knowledge, previously there is limited evidence on determinants of recommended ANC visits in Ethiopia using this advanced robust statistical method. Besides, unlike that of pocket studies in Ethiopia [23–25] at different sub regions, this study provides policy level understanding of determinants of recommended ANC visit through analysis of data with national coverage. Therefore, we aimed to assess determinants of recommended antenatal care visits in Ethiopia through mixed effects modeling. This study produced valuable evidence for policy makers and program designers working on maternal and child health by supplementing and filling the gaps in the existing body of literatures.

## Method

### Data source, study design and setting

This study analyzed data from the 2019 Mini–Ethiopian Demographic and Health Survey (MEDHS) which is part of the worldwide MEASURE DHS project. Data was downloaded from the Measure DHS website through reasonable request after data use permission was fully guaranteed.

### Sample size and sampling procedure

The Mini Ethiopian Demographic and Health Survey program (EDHS) had collected data on national representative samples of all age groups and key indicators including ANC utilization. The information on the sociodemographic, socioeconomic, and maternal-related variables was also included in the survey.

A stratified two-stage cluster sampling procedure was employed to select study participants. In the 2019 MEDHS survey, a total of 305 EAs (93 urban and 212 rural) were selected. From these enumeration areas, 149,093 households and from those households a total of 8885 reproductive-age women were included in the survey. The relevant information on the sampling procedure and data quality can be accessed elsewhere [9]. For the current study, a total of 3916 pregnant women/who gave birth in 5 years preceding the Mini Ethiopian demographic and health survey 2019 were included. The sampling weight was applied during the analysis to produce reliable estimates [26].

### Dependent variable

The dependent variable for this study was recommended ANC visits which was defined as having at list four ANC visits during pregnancy. It was coded “1” for a woman who had four and above antenatal care visits,otherwise “0” [27].

### Independent variables

After reviewing literature, educational status of mother (no formal education, primary, secondary and higher), maternal age (15–24, 25–29,30-34,35-39,40–49), parity (primipara, multipara, grand multipara), wealth status (poor, middle, rich), number of children, birth order, contraceptive utilization, media exposure (no, yes), place of residency (urban, rural) and the region which was categorized into urban (Addis Ababa, Dire Dawa, Harari), agrarian (Tigray, Amhara, Oromia and south nation nationality and peoples region) and pastoral (Somali, Afar, Gambela and Benishangul Gumuz) were considered as determinants of recommended ANC visits.

### Data management and method of analysis

Data Extraction, recoding, and both descriptive and analytical analysis were carried out using STATA version 14 software. Weighting was done to restore the representativeness of the sample. Descriptive analysis was conducted and frequencies with percentages were reported. The Generalized mixed-effects analysis was fitted after checking the intracluster correlation coefficient to adjust for random effects and produce reliable estimates. Nonlinear mixed effects modeling (mixed effects logistic regression model) was employed since the dependent variable had binary outcome.

The odds ratio was used to estimate the association between the fixed effects and the likelihood of recommended ANC visits which were expressed at a 95% confidence level. Regarding the measures of variation (random effects) intracluster correlation coefficient (ICC) and median odds ratio were reported.

## Results

### Sociodemographic characteristics of study participants

In this study, a total of 3916 women who gave birth 5 years preceding the MEDHS were included. More than half of (51.33%) of respondents had no formal education. The majority (63.70%) of respondents were exposed to media and nearly half (50.39%) of them were from poor households. Moreover, about 93.85 and 74% of participants were married and rural dwellers respectively. The majority of (55%) respondents didn’t use any contraceptive methods (Table 1).

**Table 1:** Sociodemographic characteristics of study participants, MEDHS 2019

Variables	Weighted Frequency (n)	Percentage (10%)
Maternal age		
15–24	994	25.39
25–29	1190	30.39
30–34	797	20.33
35–39	589	15.04
40–49	346	8.85
Maternal education		
No formal education	2010	51.33
Primary education	1410	36.02
Secondary and above	496	12.65
Wealth status		
Poor	1644	42.01
Middle	762	19.44
Rich	1510	38.56
Media exposure		
Yes	1421	36.30
No	2495	63.70
Parity		
Primiparous	825	21.05
Multiparous	1733	44.26
Grand multiparous	1358	34.69
Number of children		
No child	158	4.05
One child	2013	51.40
Two children	1418	36.20
Three children	327	8.35
Birth order		
First	824	21.05
2-4th	1733	44.26
≥ 5th	1359	34.69
History of contraceptive use		
No	2187	55.84
Yes	1729	44.16
Marital status		
Single	240	6.15
Married	3675	93.85
Place of residence		
Urban	1019	26.04
Rural	2896	73.96
Region		
Agrarian	3428	87.53
Pastoral	312	7.97
Urban	176	4.50
having ANC visit		
No	1003	25.62
Yes	2913	74.38

*ANC* antenatal care

### Random effect analysis

In the null model, variance component analysis was performed to decompose the total variance of recommended antenatal care visits. The applicability of mixed effects analysis instead of the traditional logistic regression model was justified by the significance of the community variance [community variance = 3.06; standard error (SE) = 0.31; *P*-value = 0.001) and intracluster correlation coefficient (ICC). The ICC in the null model indicated that about 49% of the variation of recommended ANC visits was attributed to the random effects which need to be adjusted during modeling. Moreover, the MOR was 5.25 (MOR = 5.25, 95%CI 4.48–11.70) which implied that the odds of utilizing recommended ANC visit 5.25 times higher when mothers moved from high-risk communities to low-risk ones (Table 2).

**Table 2:** Mixed effect analysis results of recommended ANC utilization in Ethiopia, MEDHS 2019

Fixed effects	Four or more ANC visits		COR 95%(CI)	AOR(95%CI)
	No	Yes		
Maternal age				
15–24	237	757	1.00	1.00
25–29	245	603	1.12(0.60–1.40)	1.83(0.77–2.64)
30–34	197	603	1.22(0.85–1.84)	1,78(0.70–2.91)
35–39	181	408	1.17(0.79–1.99)	1.71(0.98–2.90)
40–49	143	203	0.50(0.32–1.34)	0.93(0.52–1.69)
Maternal education				
No formal education	732	1278	1.00	1.00
Primary education	261	1149	2.23(1.81, 2.76)	1.55(1.22–2.01) ^a^
Secondary and above	11	495	12.01(7.24–20.27)	5.12(2.80–8.16) ^a^
Wealth status				
Poor	661	984	1.00	1.00
Middle	172	588	2.07(1.57–2.73)	1.25(1.01–1.71) ^b^
Rich	170	1340	5.06(3.75–6.82)	1.54 (1.12–2.25) ^a^
Media exposure				
Yes	167	1255	2.18(1.73–2.75)	1.23 (1.01–1.57) ^b^
No	836	1658	1.00	1.00
Parity				
Primiparous	136	688	1.00	1.00
Multiparous	368	1365	0.96(0.74–1.23)	1.14(0.70–1.52)
Grand multiparous	499	860	0.54(0.41–0.71)	0.80(0.48–1.39)
Number of children				
No child	58	101	1.00	1.00
One child	397	1616	2.08(1.37–3.18)	1.27(0.12–1.89)
Two children	398	1019	1.83(1.20–2.81)	1.58(0.78–2.43)
Three children	150	177	1.38(0.86–2.23)	1.29(0.76–2.17)
Birth order				
First	136	688	1.00	1.00
2–4	368	1365	0.96(0.74–1.23)	0.88(0.54–1.56)
≥ 5	499	860	0.54(0.41–0.71)	0.36(0.53–1.39)
History of contraceptive use				
No	760	1457	1.00	1.00
Yes	273	1456	2.37(1.90–2.97)	1.45(1.25–2.03) ^a^
Marital status				
Single	73	167	0.65(0.46–0.91)	0.75(0.59–1.23)
Married	930	2745	1.00	1.00
Place of residence				
Urban	155	865	1.00	1.00
Rural	848	2048	0.14(0.08–0.23)	0.88(0.55–1.39)
Region				
Agrarian	813	2615	1.00	1.00
Pastoral	178	134	0.22(0.13–0.37)	0.45(0.30–1.54)
Urban	12	164	1.77(1.08–2.90)	0.73(0.48–1.09)
**Random effects**				
Community variance (SE)		3.06(0.31)		
ICC (95%CI)		0.49 (0.41,0 .56)		
MOR(95%CI)		5.25(4.48,11.70)		

*ICC* intracluster correlation coefficient, *MOR* median odds ratio

^**a**^significant at < 0.05

^**b**^significant at < 0.01

### Factors associated with recommended ANC utilization

In the mixed-effects logistic regression analysis, educational status, media exposure, wealth status, and contraceptive use were significantly associated with recommended ANC visits (*p* < 0.05).

The odds of having recommended ANC visits among women with primary and above primary education was 1.55 (AOR = 1.55, 95%CI 1.22–2.01) and 5.12 (AOR = 5.12, 95%CI 2.80–8.16) respectively times higher as compared to women with no formal education. Women from households with middle and rich wealth index had 25% (AOR = 1.25, 95%CI 1.01–1.71) and 54% (AOR = 1.54, 95%CI 1.12–2.25) increased odds of having recommended ANC visits as compared to those women from poor households. The likelihood of recommended ANC visits among women who were exposed to media was 1.23 (AOR = 1.23,95%CI 1.01–1.57) times higher as compared to unexposed women. The odds of having recommended ANC visits among women who had history of contraceptive use was increased by 45% (AOR = 1.45 95%CI 1.25–2.03) as compared to women who didn’t have history of contraceptive use (Table 2).

## Discussion

This study aimed to assess the association between demographic, socioeconomic, and health care access-related factors with recommended ANC visits in Ethiopia. The odds of having recommended ANC visits among educated women was higher as compared to women with no formal education. This finding was supported by studies done in Nepal [28], East Africa [29] and Ethiopia [11, 30]. The possible explanation might be due to that educated women mostly live in urban Areas which helps them to easily access health institutions for service utilization [31]. Besides, women’s education helps to develop economic and decision-making power which will in turn improve maternal health service utilization [32].

Similarly, women from households with middle and rich wealth index had increased odds of having recommended ANC visits as compared to those women from poor households. This finding was similar to studies done in Georgia [33], India [34] and Ghana [15]. This might be due to the difficulty that women in poor households face to handle transportation and other healthcare-seeking costs [35]. Women with low economic status commonly show poor health care-seeking behavior and then poor health outcomes [36].

The likelihood of having recommended ANC visits among women who were exposed to media was higher as compared to unexposed women. This finding was consistent with studies done in Nepal [28], Bangladesh [37], Uganda [38] and Ethiopia [30]. This might be due to that media has a positive impact on safe motherhood for giving health promotion. Media also helps to develop health-seeking behavior and health care service utilization of women [39].

History of contraceptive utilization is also an important determinant of recommended ANC visit. The odds of recommended ANC visits among women with history of contraceptive use was increased as compared to women who didn’t use any contraceptive methods. This finding was similar to studies done in Tajikistan [40], Liberia [41] and Ethiopia [11]. The reason might be that the integration of family planning and other maternal health services might have given women an increased chance to have good awareness about ANC visits [42]. It might have also provided an opportunity for counseling which could avoid social barriers and encourage the ANC service utilization [38]. Besides, women’s contraceptive choice and utilization increases women’s autonomy in health-care-seeking decisions [43].

The strength of this study was that it applied the sampling weight to produce reliable estimates and used advanced model for analysis. However, due to the cross-sectional nature of the data temporal relationship between explanatory and outcome variable couldn’t be established.

## Conclusion

In this study, different factors like maternal educational status, media exposure, wealth index and history of contraceptive use were significantly associated with recommended ANC visits in Ethiopia. Therefore, encouraging women for contraceptive service utilization and consulting them to access media and improving women’s wealth status through economic and social empowerment will help to enable them to have recommended ANC visits during pregnancy in Ethiopia.

## Data Availability

All relevant data are available and not owned by third body. The dataset analyzed during the current study is available from the corresponding author on reasonable request.

## Abbreviations

ANC: Antenatal Care
AOR: Adjusted Odds Ratio
CSA: Central Statistical Agency
EAs: Enumeration Areas
MEDHS: Mini Ethiopia Demographic and Health Survey
SNNP: South Nation Nationality and People
WHO: World Health Organization
